# Contrast-Enhanced Ultrasound-Magnetic Resonance Imaging Radiomics Based Model for Predicting the Biochemical Recurrence of Prostate Cancer: A Feasibility Study

**DOI:** 10.1155/2022/8090529

**Published:** 2022-04-28

**Authors:** Yong Wang, Guoyan Feng, Jianru Wang, Peng An, Peng Duan, Yan Hu, Yingjian Ye, Yang Li, Ping Qin, Ping Song

**Affiliations:** ^1^Department of Radiology, Xiangyang No. 1 People's Hospital, Hubei University of Medicine, Xiangyang 441000, China; ^2^Department of Internal Medicine, Xiangyang No. 1 People's Hospital, Hubei University of Medicine, Xiangyang 441000, China; ^3^Department of Reproductive Medicine, Xiangyang No. 1 People's Hospital, Hubei University of Medicine, Xiangyang 441000, China; ^4^Department of Radiology, The Affiliated Hospital of Nanjing University of Chinese Medicine, Jiangsu Province Hospital of Chinese Medicine, The First Clinical Medical College, 155 Hanzhong Road, Nanjing, 210029 Jiangsu Province, China; ^5^Department of Pharmacy and Laboratory, Xiangyang No. 1 People's Hospital, Hubei University of Medicine, Xiangyang 441000, China

## Abstract

**Objective:**

This study was aimed at developing a model for predicting postoperative biochemical recurrence of prostate cancer (PCa) using clinical data-CEUS-MRI radiomics and at verifying its clinical effectiveness.

**Methods:**

The clinical imaging data of 159 patients pathologically confirmed with PCa and who underwent radical prostatectomy in Xiangyang No. 1 People's Hospital and Jiangsu Hospital of Chinese Medicine from March 2016 to December 2020 were retrospectively analyzed. According to the 2-5-year follow-up results, the patients were divided into the biochemical recurrence (BCR) group (*n* = 59) and the control group (*n* = 100). The training set and test set were established in the proportion of 7/3; 4 prediction models were established based on the clinical imaging data. In training set, the area under the curve (AUC) and decision curve analysis (DCA) by R was conducted to compare the efficiency of 4 prediction models, and then, external validation was performed using the test set. Finally, a nomogram tool for predicting BCR was developed.

**Results:**

Univariate regression analysis confirmed that the SmallAreaHighGrayLevelEmphasis, RunVariance, Contrast, tumor diameter, clinical T stage, lymph node metastasis, distant metastasis, Gleason score, preoperative PSA, treatment method, CEUS-peak intensity (PI), time to peak (TTP), arrival time (AT), and elastography grade were the influencing factors for predicting BCR. In the training set, the AUC of combinatorial model demonstrated the highest efficiency in predicting BCR [AUC: 0.914 (OR 0.0305, 95% CI: 0.854-0.974)] vs. the general clinical data model, the CEUS model, and the MRI radiomics model. The DCA confirmed the largest net benefits of the combinatorial model. The test set validation gave consistent results. The nomogram tool has been well applied clinically.

**Conclusion:**

The previous clinical and imaging data alone did not perform well for predicting BCR. Our combinatorial model firstly using clinical data-CEUS-MRI radiomics provided an opportunity for clinical screening of BCR and help improve its prognosis.

## 1. Introduction

With the acceleration of China's industrialization process and the impact of environmental pollution, the incidence of prostate cancer (PCa) caused by enriched food, smoking, excessive alcohol use, and alcoholism keeps rising, with a value of 6.63% increase per year. According to literature, the recurrence rate of PCa within 3-5 years after treatment is around 28-34%, mostly presented increased serum prostate-specific antigen (PSA), that is, biochemical recurrence (BCR) [1, 2]. Currently, the American Urological Association (AUA) guidelines consider biochemical recurrence (with PSA ≥ 0.2 ng/mL for two consecutive follow-up tests) as a precursor of clinical recurrence of PCa. In the absence of effective medical intervention, about 36% of patients would transform into clinical recurrence, even with bone metastasis, in 12-36 months after BCR [3, 4]. PCa patients in China are generally 65+ years old; many patients and even doctors believe that prostate cancer had a good prognosis just like thyroid cancer due to the lack of medical knowledge by patients, the insensitivity of PSA test reagents, and the incomprehension of PCa guidelines by doctors. Frequent follow-up checks are considered tedious, and the comprehensive surveillance and follow-up of BCR are difficult in practice. Therefore, the selection of BCR target population is critical. It has been reported that the clinical stage of PCa, PSA level, radical treatment method, and Gleason score were the risk factors for BCR in PCa patients. Murata et al. reported 90% biochemical recurrence in 24 months after surgery for patients with more than three BCR-related risk factors above. However, Farkas et al. believed that the false-positive rate of BCR was 30%. Our team have similar findings too, indicating that these risk factors were poor predictors of BCR [4, 5]. Therefore, the development of new predictive models for patients with large individual differences is extremely important, but studies in this area have rarely been reported. Our team has read lots of literatures on BCR. Many studies' contents are relatively single and do not evaluate the diagnostic differences of various imaging technologies. Moreover, valuable imaging texture parameters cannot be deeply mined to predict BCR. Hence, our team adopted contrast-enhanced ultrasound (CEUS) combined with magnetic resonance imaging (MRI) radiomics and clinical data to establish several models/a nomogram tool to predict BCR and achieved good results, providing an opportunity for clinically accurate assessment of BCR for individually different patients (Figures 1 and 2).

## 2. Materials and Methods

### 2.1. Inclusion and Exclusion Criteria

The clinical and imaging data of 159 patients diagnosed with PCa by CEUS-guided prostate biopsy or postoperative pathological examination in Xiangyang No. 1 People's Hospital and Jiangsu Hospital of Chinese Medicine from March 2016 to December 2020 were retrospectively analyzed. The enrolled patients were between 63 and 91 years old, with a mean age of 72.6 ± 16.7. The inclusion criteria were (1) following the PCa diagnostic criteria of the European Association of Urology and the American Urological Association; (2) only single lesions visible by MRI and ultrasound were studied in order to reduce research bias; (3) patients with untreated primary prostate cancer; and (4) patients with complete clinical imaging data, good compliance, and long follow-up period. The exclusion criteria were as follows: (1) patients with tumors involving other organs; (2) patients with congenital heart disease, heart failure, liver and kidney insufficiency, history of allergies, and contraindications to enhanced imaging; and (3) patients with cognitive impairment [2, 6]. This study has obtained the signed informed consents from the patients or their families and was approved by the Ethics Committee of Xiangyang No. 1 People's Hospital and Jiangsu Hospital of Chinese Medicine.

### 2.2. Research Methods

#### 2.2.1. Clinical History Data

The clinical history data included laboratory parameters, age, prostate volume, tumor diameter, BMI, clinical T stage, lymph node metastasis, distant metastasis, Gleason score, preoperative PSA, and treatment mode.

#### 2.2.2. Magnetic Resonance Imaging

The Philips Achieva SE 1.5T Signa HD and Siemens Avanto Class 1.5T MRI scanner (Netherlands Eindhoven-Amsterdam United Company& Siemens medical Corporate Technology, Germany) equipped 6-channel phased array body coils with updated multi sequence scanning parameters system 4.0.3 were selected. The patient was required in a supine posture. The midlower abdomen/pelvis including prostate, bladder, and surrounding tissues were first covered, followed by scanning range from ≥2 cm above the bottom of the bladder to the external genitalia. Then, the transverse, sagittal, and coronal T2WI and the sagittal T1WI images of the bladder and prostate were stored. The T2WI images were obtained using single-shot fast spin echo (SSTSE) and balanced steady-state free precession gradient echo sequences (balance FFE). The SSTSE parameters included TR 7,500 ms, TE 110 ms, flip angle 90°, matrix 350 × 350, slice thickness 2-5 mm, and field of view (FOV) 25 × 25 cm. The balance FFE parameters included TR 3.50 ms, TE 1.5 ms, flip angle 90°, and slice thickness 3-8 mm. DWI (diffusion-weighted imaging) and ADC (apparent diffusion coefficient) were obtained with reference to conventional sequences. The T1WI was acquired by breath-holding fast spin echo sequence (FSE) using the following variable parameters: TR 850 ms, TE 10-15 ms, matrix 250 × 250, slice thickness 2-5 mm, and FOV 25 × 25 cm [7, 8].

#### 2.2.3. Radiomics Analysis

The 3D slicer (Version 4.11.20210226, https://www.slicer.org/) image segmentation software was used to delineate the region of interest (ROI) of magnetic resonance images, and then, texture analysis and data extraction were conducted. After determining the candidate texture data such as firstorder, glcm, shape, and ngtdm, R X64 (Version 4.1.3, the R Project for Statistical Computing, version 4.1.3, https://www.r-project.org/) was used to carry out Lasso regression analysis to extract valid texture data from the candidate texture data [8].

#### 2.2.4. CEUS Procedure

The Mindray-Resona R9 and GE LOGIQ E9 (U.S.) ultrasound scanners were adopted, using the broadband transrectal convex array transducer (frequency range 4.5-9.5 MHz). After the patient did enema cleaning, the probe was covered with a medical condom or probe cover and inserted into the patient's rectum. First, the routine examination of the prostate through rectum was performed in which the density distribution and blood flow signals of the prostate were observed, and the size of the prostate and the diameter of the tumor were measured. With no sign of patient discomfort, SonoVue, an ultrasound contrast agent from Bracco (Italy), was injected. The section with the largest cross-sectional area of the lesion was taken as the base point, and the observation direction was frequently adjusted. A volume of 2.4-3.0 mL of contrast agent was pulsed injected through the median cubital vein and then flushed quickly with 5-15 mL of 9 mg/mL sodium chloride solution. The real-time enhancement was monitored and recorded during pulsed injection. After 3-5 min, the raw DICOM images and videos were stored in the Neusoft PACS system. Then, TIC (time-intensity curve), the analysis software, was used to record the peak intensity (PI), ascending branch slope (*Σ*), descending branch slope (*γ*), time to peak (TTP), arrival time (AT), and area under the curve (AUC) of the time-intensity curve of ROI. All examinations were carried out independently by the two deputy chief sonographers. For any disagreement, it was resolved by consulting and discussing with a third independent senior sonographer [9].

#### 2.2.5. Grading of Pathological Materials

A number of 3-6 pieces of biopsy specimens were taken from the patient's rectal ultrasound and sent for pathological examination. The Gleason grading was performed after the diagnosis of PCa.

#### 2.2.6. Radical Prostatectomy for PCa

Under general anesthesia, the patient's posterior of the prostate and rectum was separated to expose the apex of the prostate, the anterior bladder space, and the retropubic space. After prostatectomy, the bladder neck reconstruction and urethral anastomosis were conducted.

#### 2.2.7. Endocrine Therapy

Conventional medical castration using luteinizing hormone-releasing hormone (LH-RH) analogues was conducted, together with antiandrogen or testicular surgery followed by goserelin+bicalutamide [10, 11].

#### 2.2.8. Follow-Up Observation and Prognosis

After the operation, the patients were asked to check the PSA levels regularly in the outpatient department. In the first two years after surgery, the PSA check and follow-up should be performed one month after the operation and every three months afterwards. After two years, the PSA check and follow-up should be performed every six months, and MRI should be conducted when necessary. During the follow-up period, the cases with elevated PSA levels of ≥0.2 ng/mL for two or more consecutive follow-up tests were included in the study group (the biochemical recurrence group), and the others were included in the control group.

### 2.3. Statistical Methods

All statistical analyses were carried out using the R version 4.1.3 (R Foundation for Statistical Computing, version 4.1.3; https://www.r-project.org/). The independent samples *t*-test or the *χ*^2^ test or Fisher's exact test was applied for intergroup comparisons following data normal distribution test (*P* < 0.05). And then, 4 prediction models, decision curves, and nomograms were established by logistic regression or R software 4.1.3 using the above-mentioned risk factors in the training set. Then, the modified combined models were validated using test set. The larger AUC, the higher prediction with the *P* value < 0.05 (two-tailed) confirmed statistical significance. Other statistical software was the SPSS 22.0 (IBM SPSS Statistics GradPack and Faculty Packs, USA; https://www.ibm.com/products/spss-statistics) [10, 12].

## 3. Results

### 3.1. Follow-Up Results

At the end of the follow-up period, six of the 181 PCa patients were lost to follow-up, five refused follow-up, and 11 had other tumors or liver and kidney insufficiency. A total of 59 patients were clinically diagnosed with BCR (the study group), and 100 patients were BCR-free for 24-48 months (the control group). The 2-5-year BCR rate of PCa patients was 37.11% (59/159) (Figure 3).

### 3.2. Data Extraction

Our team extracted a total of 874 sets of texture data based on the prostate cancer ROI delineated by 3D slicer and then screened out a total of 14 sets of useful data based on the Lasso regression conducted by R. After normal distribution test and independent sample *t*-test, three sets of effective data were finally obtained, the gray-level size zone matrix (SmallAreaHighGrayLevelEmphasis and RunVariance) and the neighborhood gray-tone difference matrix (Contrast) (Figure 4 and Table 1).

### 3.3. Comparative Analysis of Clinical CEUS Characteristics of PCa Patients between the Study Group and the Control Group

Univariate analysis demonstrated that in the study group, clinical T stage, lymph node metastasis or distant metastasis, tumor size, Gleason score, preoperative PSA level, treatment method, TTP, PI, and AT of the time-intensity curve of CEUS were significantly higher/lower than those of the control group (*P* < 0.05) (Tables 2 and 3).

### 3.4. Multivariate Analysis of Biochemical Recurrence of PCa after Treatment

Multivariate logistic regression analysis showed that Gleason score, preoperative PSA level, treatment method, elastography grade, and gray-level size zone matrix (SmallAreaHighGrayLevelEmphasis and RunVariance) were the independent risk factors for biochemical recurrence of PCa after surgery (all *P* < 0.05) (Table 4).

### 3.5. Establishment of Multiple Predictive Models and External Validation

Based on the above risk factors, a variety of predictive models (the general data model, CEUS model, MRI radiomics model, and combinatorial model) were established using R in the training set. The MedCalc (Version 20.0.22) was used to compare their predictive performance. The results demonstrated that the combinatorial model was superior regarding the predictive value, with an AUC of 0.914 (OR 0.0305, 95% CI: 0.854-0.974), significantly higher than the general data model [AUC: 0.769 (OR 0.0480, 95% CI: 0.675-0.863), *P* = 0.0008], CEUS model [AUC: 0.783 (OR 0.0461, 95% CI: 0.692-0.873), *P* = 0.0035], and MRI radiomics model [AUC: 0.730 (OR 0.0513, 95% CI: 0.629-0.830), *P* = 0.0002]. The subsequent decision curve analysis conducted by R also confirmed that the net benefit of the combinatorial model was significantly higher than the other models. Finally, the expected results were also verified in the test set. The combinatorial model exhibited the highest predictive performance [AUC: 0.920 (OR 0.0362, 95% CI: 0.849-0.991])], significantly higher than the general data model [AUC: 0.716 (OR 0.0701, 95% CI: 0.578-0.853), *P* = 0.0007], CEUS model [AUC: 0.814 (OR 0.0533, 95% CI: 0.709-0.918), *P* = 0.0461], and MRI radiomics model [AUC: 0.764 (OR 0.0621, 95% CI: 0.642-0.885), *P* = 0.0109] (Figures 5 and 6).

The nomogram tool and calibration curve of biochemical recurrence of PCa patients were made by R and then applied clinically (Figure 7).

## 4. Discussion

According to the World Health Organization (WHO) data, in European and American countries, 230,000 to 250,000 males are diagnosed with prostate cancer every year. About 40% of PCa patients underwent radical prostatectomy. Although the overall success rates for localized prostate cancer control were high clinically, 20-30% of patients experienced biochemical or clinical recurrence, which initially presented as elevated PSA without specific clinical distant or radiographic metastases. The biochemical recurrence shows the presence of residual prostate epithelial tissue in the body and is thought to indicate cancer [11, 12]. In addition, the clinical course of PCa patients varied a lot. Some patients experienced rapid disease progression to metastasis, while a small number of patients had long-term survival because of activated immune system accompanying PSA fluctuations, but with shortened life expectancy. And in rare cases, no survival impact was observed. Therefore, for PCa patients, the postoperative PSA levels should be closely monitored. It has been reported that the early diagnosis of biochemical recurrence and effective medical intervention could significantly prevent or reduce the incidence of clinical recurrence of PCa and metastasis [13, 14]. In this study, the prediction tool based on clinical-CEUS-MRI radiomics parameters achieved better prediction outcomes, and the combinatorial model based on the above influencing factors was also dramatically better than the other models.

The PubMed database has few studies (<20 articles) on the prediction of biochemical recurrence of PCa based on ultrasound combined with MRI, while the studies on biochemical recurrence based on radiomics were barely reported. This study followed up the medical records of 159 patients with PCa in Xiangyang No. 1 People's Hospital and Jiangsu Hospital of Chinese Medicine. The results showed that the BCR rate of PCa within 2-5 years was as high as 37.11%, slightly higher than the data reported by post JM. Presumably, it is because that this study was a single-center study with a short follow-up period. Therefore, it is necessary to closely follow up the prognosis of patients after radical prostatectomy and build a model for early prediction of biochemical recurrence of PCa. In order to dig out effective parameters for accurate prediction of the biochemical recurrence of PCa, our team firstly compared the clinical history-CEUS-MRI radiomics data between the study group and the control group. Then, the univariate regression results demonstrated significant differences between the two groups (*P* < 0.05) regarding clinical T staging, lymph node/distant metastasis, tumor size, Gleason score, preoperative PSA level, treatment method, PI and AT of the time-intensity curve of CEUS, the gray-level size zone matrix (SmallAreaHighGrayLevelEmphasis and RunVariance), and the neighborhood gray-tone difference matrix (Contrast) from radiomics. The binary logistic regression analysis confirmed that Gleason score, preoperative PSA level, treatment method, and gray-level size zone matrix (SmallAreaHighGrayLevelEmphasis and RunVariance) were independent risk factors for biochemical recurrence of PCa. It was suggested that the tumor volume and CEUS arrival time, etc., would perform poorly on independent predication of the biochemical recurrence of PCa. It has been reported that the treatment method, Gleason score, preoperative PSA level, and distant lymph node metastasis were known important factors for the biochemical recurrence of PCa. However, in this study, the independent prediction performances of the above factors were poor. Furthermore, it was unable to provide effective early warning for patients with large individual differences, which was also related to the evolution of the disease. Preoperative PSA level was an available quantitative indicator, but with poor specificity. It was easily affected by reagent sensitivity, age, and other diseases (such as urinary infection, prostatitis, and endocrine and metabolic diseases); therefore, PSA was a weak independent predictor of biochemical recurrence of PCa [15–17].

From a statistical point of view, many indicators in CEUS-elastography displayed large comparative differences in sample size, and they may serve as effective indicators for predicting biochemical recurrence. In particular, it was revealed in this study that the rapid enhancement in the arterial phase of the study group was significantly higher than that of the surrounding normal prostate area. Therefore, it may be a potential indicator for predicting biochemical recurrence. In addition, the TTP of the study group was significantly smaller than that of the control group, whereas the PI was significantly larger than that of the control group (both *P* < 0.05). These may be related to the rich blood supply and the low tumor differentiation of PCa in the study group, similar to those reported in the literature [18, 19]. The concept of radiomics was first proposed by the Dutch scholar Lambin in 2012 and was first applied to X-ray, and computer vision is dramatically better than human vision. At present, the 3D slicer and ITK-snap software developed by Harvard University and others have extended the concept of omics to ultrasound, computed tomography (CT), MRI, and pathology. In the past decade, various high impact factor and high-quality omics studies have sprung up rapidly like bamboo shoots after the rain. Therefore, in the study of PCa biochemical recurrence, we also introduced radiomics parameters and achieved good outcomes. After delineating the ROI of preoperative MRI data of the 159 PCa cases and screening, we extracted a total of three sets of reliable radiomics data, the gray-level size zone matrix (SmallAreaHighGrayLevelEmphasis and RunVariance) and the neighborhood gray-tone difference matrix (Contrast). These data represented the signal intensity and density of the lesion and gradient variance, respectively. Our team then constructed four prediction models based on all the above-mentioned risk factors and chose a training set and a test set for training verification and obtained consistent results. Finally, based on DeLong nonparametric and the decision curve analysis, it was confirmed that the combinatorial model had a good prediction outcome, with AUC significantly higher than the other models. The developed nomogram prediction tool has also been well applied clinically. This may be because that this nomogram prediction tool combined the clinical-CEUS-MRI radiomics indicators and then obtained PCa patient-based individualized parameters, thereby improving the accuracy of prediction [20, 21]. The combinatorial model is helpful for early prediction of biochemical recurrence and early adjustment of intervention and treatment plans in clinical practice, suppressing the malignant progression of biochemical recurrence and improving the quality of life and survival rate of patients.

## 5. Limitations

The data size of this study was small. In the future, multicenter studies involving multiple hospitals will be needed. This study also lacked pathomics studies and lacked radiomics extraction based on CEUS results; therefore, the mining of ultrasound-pathology data was not deep enough. In addition, predictive models have been widely used in clinical research and risk decision-making but based on the strict linear relationship and normal distribution of data. In order to solve these limitations, our team will use advanced machine learning algorithms (XGboost, LightGBM, or CatBoost) to establish an ensemble modeling in the future to further improve the prediction accuracy. And we will conduct multicenter research to verify our prediction tools [22].

## 6. Conclusion

In conclusion, the combined model established based on clinical-CEUS-MRI parameters provided a better opportunity for predicting biochemical recurrence in PCa patients, and it can also serve as a basis for early adjustment of interventional treatment plans for individualized clinical cases.

## Figures and Tables

**Figure 1:** From the content of references retrieval from 1980 to 2021, BCR has always been a research hotspot, with more research on molecular mechanism and BCR management and but less on prediction of BCR by multimodal radiomics.

**Figure 2:** The technical flowchart of this study. Novelty of the work is a prediction model/nomograph tools established using the multimodal radiomics (MRI-ultrasound) combined with clinical data, which has not been reported before.

**Figure 3:** The simplified inclusion and exclusion criteria for patient enrollment in the present study.

**Figure 4:** Schematic diagram of texture omics feature extraction based on R Studio software (lasso regression method of deep learning). A total of 14 groups of available texture data are extracted.

**Figure 5:** DeLong nonparametric method was used to estimate the area under the curve of ROC between different prediction models of training set (a) and test set (b) and compare its effectiveness in predicting the BCR. The area under the curve of the combined model was the largest.

**Figure 6:** In the training set (a) and the test set (b), the prediction performance of the general data model, CEUS model, MRI radiomics model, and combinatorial model is compared using the net benefit of decision curve; it is confirmed that the combined model had the highest predictive performance.

**Figure 7:** The nomogram prediction tool based on the risk factors of the combined model was used clinically (x5 Gleason score; X6 preoperative PSA concentration; X7 treatment mode; X11 elastography grade; x12 SmallAreaHighGrayLevelEmphasis; and x13 RunVariance).

**Table 1:** Regression analysis results of establishing MRI model based on MRI radiomics to predict the BCR, ^∗^*P* < 0.05.

MRI radiomics model	Univariate analysis		Multivariate analysis	
	*P*	Hazard ratio	*P*	Hazard ratio
Median...86	0.247	0.714 (0.404-1.262)		
DifferenceVariance...105	0.754	0.962 (0.758-1.223)		
SmallDependenceEmphasis...133	0.637	1.067 (0.815-1.396)		
DifferenceAverage...227	0.123	1.274 (0.937-1.731)		
SumEntropy...240	0.061	1.299(0.989-1.708)		
SmallDependenceHighGrayLevelEmphasis...321	0.293	0.632 (0.268-1.488)		
Maximum...329	0.645	1.081 (0.776-1.506)		
Variance...338	0.495	1.231 (0.678-2.237)		
Idm...350	0.797	1.017 (0.896-1.154)		
InverseVariance...354	0.695	1.031 (0.887-1.201)		
SmallAreaHighGrayLevelEmphasis...665	0.045^∗^	1.322 (1.006-1.737)	.021^∗^	1.418 (1.054-1.906)
RunVariance...758	0.021^∗^	0.484 (0.262-0.897)	.017^∗^	0.443 (0.227-0.865)
Contrast...866	0.047^∗^	0.772 (0.598-0.996)	.034^∗^	0.748 (0.571-0.979)
Strength...872	0.366	1.068 (0.926-1.231)		

**Table 2:** Regression analysis results of establishing general data model based on clinical features to predict the BCR, ^∗^*P* < 0.05.

General data model	Univariate analysis		Multivariate analysis	
	*P*	Hazard ratio	*P*	Hazard ratio
Age (year)	0.549	1.027 (0.941-1.123)		
Prostate volume (cm^3^)	0.772	0.994 (0.956-1.034)		
Tumor diameter (mm)	0.038^∗^	1.431 (1.021-2.003)	0.081	1.441 (0.956-2.174)
BMI (kg/m^2^)	0.815	0.985 (0.869-1.117)		
Clinical T stage	0.027^∗^	1.839 (1.071-3.159)	0.219	1.518 (0.781-2.953)
Lymph node metastasis	0.017^∗^	1.469 (1.072-2.013)	0.027^∗^	1.526 (1.049-2.221)
Distant metastasis	0.041^∗^	1.404 (1.015-1.942)	0.621	1.107 (0.739-1.659)
Gleason score	0.049^∗^	2.331 (1.004-5.409)	0.050	2.788 (0.998-7.788)
Preoperative PSA (*μ*g/L)	0.031^∗^	2.248 (1.075-4.701)	0.035^∗^	2.571 (1.070-6.178)
Treatment mode	0.022^∗^	2.667 (1.152-6.172)	0.022^∗^	3.263 (1.189-8.955)

**Table 3:** Regression analysis results of establishing CEUS model based on CEUS features to predict the BCR, ^∗^*P* < 0.05.

CEUS model	Univariate analysis		Multivariate analysis	
	*P*	Hazard ratio	*P*	Hazard ratio
PI (dB)	0.025^∗^	0.794 (0.648-0.971)	0.083	0.827 (0.667-1.025)
*Σ*	0.395	1.441 (0.622-3.336)		
*γ*	0.533	1.308 (0.562-3.042)		
TTP	0.044^∗^	1.010 (1.000-1.019)	0.074	1.009 (0.999-1.020)
AT	0.028^∗^	1.165 (1.017-1.334)	0.079	1.144 (0.984-1.329)
AUC	0.753	0.877 (0.386-1.989)		
Enhanced level	0.872	0.934 (0.408-2.137)		
Enhanced uniformity	0.781	0.891 (0.394-2.013)		
Elastography grade	0.013^∗^	2.515 (1.218-5.191)	0.019^∗^	2.581 (1.771-5.692)

Notes: PI: the peak intensity; *Σ*: ascending branch slope; *γ*: descending branch slope; TTP: time to peak; AT: arrival time.

**Table 4:** Regression analysis results of establishing combinatorial model based on CEUS-MRI-clinical features to predict the BCR, ^∗^*P* < 0.05.

Combinatorial model	*B*	S.E.	Wals	Sig.	Exp (*B*)	Exp (*B*) 的 95% C.I.	
						Lower limit	Upper limit
SmallAreaHighGrayLevelEmphasis	.706	.248	8.144	.004^∗^	2.027	1.248	3.293
RunVariance	.913	.472	3.746	.037^∗^	.401	.159	1.012
Contrast	.360	.208	3.002	.083	.698	.464	1.048
Tumor diameter (mm)	.606	.276	4.818	.068	1.833	1.067	3.148
Clinical T stage	.086	.420	.042	.838	1.090	.479	2.482
Lymph node metastasis	.444	.262	2.873	.090	1.558	.933	2.603
Distant metastasis	.573	.320	3.201	.074	1.773	.947	3.321
Gleason score	1.245	.657	3.596	.048^∗^	3.474	.959	12.583
Preoperative PSA (*μ*g/L)	1.425	.579	6.044	.014^∗^	4.156	1.335	12.941
Treatment mode	1.580	.707	4.992	.025^∗^	4.854	1.214	19.410
PI (dB)	.177	.156	1.279	.258	.838	.617	1.138
TTP	.008	.007	1.120	.290	1.008	.994	1.022
AT	.175	.113	2.391	.122	1.191	.954	1.487
Elastography grade	1.324	.579	5.234	.022^∗^	3.757	1.209	11.675

## Data Availability

All data generated or analyzed during this study are included in this published article.
